# Development of a Portable Respiratory Gas Analyzer for Measuring Indirect Resting Energy Expenditure (REE)

**DOI:** 10.1155/2021/8870749

**Published:** 2021-02-17

**Authors:** Hyo-Chang Seo, Daehyeon Shin, Chae Hun Leem, Segyeong Joo

**Affiliations:** ^1^Department of Biomedical Engineering, Asan Medical Institute of Convergence Science and Technology, Asan Medical Center, University of Ulsan College of Medicine, Seoul, Republic of Korea; ^2^Department of Physiology, Ulsan College of Medicine, Seoul, Republic of Korea

## Abstract

**Objective:**

A rapidly growing home healthcare market has resulted in the development of many portable or wearable products. Most of these products measure, estimate, or calculate physiologic signals or parameters, such as step counts, blood pressure, or electrocardiogram. One of the most important applications in home healthcare is monitoring one's metabolic state since the change of metabolic state could reveal minor or major changes in one's health condition. A simple and noninvasive way to measure metabolism is through breath monitoring. With breath monitoring by breath gas analysis, two important indicators like the respiratory quotient (RQ) and resting energy exposure (REE) can be calculated. Therefore, we developed a portable respiratory gas analyzer for breath monitoring to monitor metabolic state, and the performance of the developed device was tested in a clinical trial. *Approach*. The subjects consisted of 40 healthy men and women. Subjects begin to measure exhalation gas using Vmax 29 for 15 minutes. After that, subjects begin to measure exhalation gas via the developed respiratory gas analyzer. Finally, the recorded data on the volume of oxygen (VO_2_), volume of carbon dioxide (VCO_2_), RQ, and REE were used to validate correlations between Vmax 29 and the developed respiratory gas analyzer.

**Results:**

The results showed that the root-mean-square errors (RMSE) values of VCO_2_, VO_2_, RQ, and REE are 0.0315, 0.0417, 0.504, and 0.127. Bland-Altman plots showed that most of the VCO_2_, VO_2_, RQ, and REE values are within 95% of the significance level.

**Conclusions:**

We have successfully developed and tested a portable respiratory gas analyzer for home healthcare. However, there are limitations of the clinical trial; the number of subjects is small in size, and the age and race of subjects are confined. The developed portable respiratory gas analyzer is a cost-efficient method for measuring metabolic state and a new application of home healthcare.

## 1. Introduction

The global home healthcare market size was valued at USD 305.78 billion in 2018 and is expected to register a Compound Annual Growth Rate (CAGR) of 7.8% over the forecast period. Since 2010, the growing market has introduced many devices for the home or wearable healthcare products [1–3]. Most of these healthcare devices measure blood pressure, heart rate, and training data, such as steps or ran/cycled distances.

A variety of portable and wearable devices have been developed and are already available on the market. Many devices have been studied, such as measuring PTT, gait speed, step count, stride time, and heart rate related to daily activities. For the PTT case, There are many research studies on the negative correlation between pulse transit time (PTT) and blood pressure (BP) [4–6]. In addition, putting an electrocardiogram (ECG) with a piezoelectric sensor on the wrist showed that measuring PTT was also possible [7]. For gait analysis, insole-type equipment was introduced and showed excellent performance in measuring basic gait parameters, such as step count and stride time [8]. A commercial device for measuring pressure distribution within a shoe with multiple pressure and acceleration sensors in the insole is currently available (Runvi, Germany). Many commercial health care products tend to record activities (i.e., heart rate) through devices worn on the wrist or around the chest, and the user can manage their data with a smartphone application or on the web (Wahoo TICKR, Wahoo Fitness, USA). Several wristwatch devices can measure ECGs, such as Apple Watch (Apple, USA), Move ECG (Withings, France), and Amazfit Verge 2 (Huami, China).

Though various portable or wearable healthcare products have already been developed and are currently available on the market, most of these products focus on measuring, estimating, or calculating physiologic signals or other parameters, such as step counts, blood pressure, and electrocardiogram. However, many of these devices cannot monitor the metabolic state. Continuous monitoring of metabolic state could reveal minor or major changes in one's health condition. Breath analysis is a simple, noninvasive way of measuring metabolism [9, 10].

Respiration is associated with biological metabolic activity [11]. Metabolism is the process of converting nutrient intake into energy for maintaining cellular homeostasis. Metabolism consists of catabolism and anabolism. Catabolism is the process of converting ingested macromolecules (i.e., food) into monomers (i.e., Triglycerides, monosaccharides) through mechanisms like hydrolysis, in order to gain all the nutrients the human body requires. Anabolism is the process of synthesizing basic molecules into more complex ones. Humans require energy to support normal metabolic functions, such as the growth and repair of tissues and draining debris, and to support physical activity. Energy is provided by the oxidation of dietary carbohydrates, fats, and proteins and is expressed as calories. Resting energy expenditure (REE) is one of the respiratory indicators that can measure the energy used by metabolic activity. REE is the amount of energy consumed by people at rest and is widely used as an indicator of their metabolism and nutritional status. Therefore, the development of a portable device for measuring REE is important for healthcare monitoring.

Another important index for measuring caloric consumption is the respiratory quotient (RQ). RQ is a dimensionless number used in the evaluation of the basal metabolic rate when estimated through carbon dioxide production. It is calculated through the body carbon dioxide production-body oxygen consumption ratio. Carbohydrates are involved in energy production when the RQ value is close to 1.0, proteins are involved when the value is close to 0.8, and fats are involved as the main energy source when the value is close to 0.7 [12–14]. Therefore, the RQ value is also important because it is related to metabolic activity.

Currently, REE and RQ are measured by using an indirect calorimeter [15]. However, commercially available indirect calorimeters are large and expensive. Furthermore, the device can be operated only by trained staff. Therefore, it is obvious that a portable and low-cost gas analyzer could help in managing one's healthcare, especially for measuring metabolic state changes.

In this paper, we developed a new portable and cost-effective gas analyzer for monitoring metabolic states in users' homes, and equivalence with the reference calorimeter through clinical trials was demonstrated.

## 2. Materials and Methods

To build a portable respiratory gas analyzer, the system needs to measure respiratory volume and the concentration of both oxygen and carbon dioxide. The measured results are displayed on a tablet PC in real time. Oxygen and carbon dioxide concentrations were measured by sampling with a DC motor. We also developed software to display and store the measured results. It is designed to be used by nonexperts. We also conducted a clinical trial to validate correlations between the developed device and a commercial device. A detailed description is provided hereinafter.

### 2.1. Respiratory Gas Analyzer Design

The functional diagram of the developed system is shown in Figure 1. The respiratory gas analyzer is composed of a flow sensor (D6F-10A5, OMRON, Japan), a CO_2_ sensor (SprintIR®-W Carbon Dioxide Sensor, CO_2_ Meter, USA), and an O_2_ sensor (MLF-350, ITG, Germany). First, a mask is used to obtain the user's respiratory parameters. When the user exhales, a flow sensor attached to the back of the mask measures the respiratory strength. The water trap is then used to remove moisture before oxygen and carbon dioxide measurements are taken, as moisture could affect the measurement. A DC motor is used to supply moisture-removed air to each sensor, and the measured values are designed to be displayed on a tablet PC in real time. The type of flow sensor is a MEMS mass flow sensor that measures the flow rate of gas by using a temperature difference. The CO_2_ sensor is a nondisruptive infrared (NDIR) sensor type, which detects the concentration of gas by measuring the degree of light absorption by the gas analyte. The O_2_ sensor is a galvanic fuel cell type, which is commonly used to measure the concentration of oxygen gas.

The flow sensor was attached to the mask to directly measure the velocity of exhalation flow. Some of the exhaled gas is extracted into the body of the respiratory gas analyzer by a DC motor to measure O_2_ and CO_2_ partial pressure. A DC motor (Diaphragm Pump 2002 VD LC, THOMAS, Germany) with a flow of 500 ml per minute and a max pressure of 400 mbar was adopted to collect the sample volume (about 5% to 10%) of the exhaled gas. Since the respiratory volume per minute is approximately 6000∼10000 ml per minute, a DC motor that met the requirements was selected. Normal tidal volume is approximately 400∼500 ml and respiratory rate per minute is about 15∼20 breaths. To prevent performance degradation of the infrared- (IR-) based CO_2_ sensor, moisture in the exhaled gas was filtered using a water trap.

The CO_2_ sensor had a response time of 50 ms and a measurement range of 0 to 20%, while the O_2_ sensor had a response time of 350 ms and a measurement range of 0 to 35%. O_2_ sensor has a lower response speed than the CO_2_ sensor, but this is enough in measuring partial pressure. The communication protocols of CO_2_ sensor, O_2_ sensor, and flow rate sensor modules are UART (baud rate of 9600), *I*^2^*C*, and analog output, respectively. To control these sensors simultaneously, a microcontroller (ATmega 128, Atmel, USA) with a built-in 12-bit analog-to-digital converter (ADC), UART, and I^2^C controller was utilized. The output of these sensors was sampled at 20 Hz and transferred to a tablet PC with a UART interface (baud rate of 115200).

The software for processing the transmitted data and displaying the measured and evaluated values through a user interface was also developed. A Windows-based tablet PC (Dell Venue 8 Pro, Dell, USA) was used, and the software was developed using LabVIEW (LabVIEW2017, National Instruments, USA). The software runs in four steps: (1) the user is required to fill out the subject's personal information, (2) each sensor is then calibrated for 30 seconds, (3) after a pause, the software automatically goes to the next step and a reminder to wear the mask pops up, and pressing the “OK” button leads to the measurement window, and (4) when the “Start” button is pressed, the measurement starts, and values are displayed on the screen in real time. The measured data is automatically stored on the tablet PC.

### 2.2. REE and RQ Calculation

REE can be calculated indirectly through the relationship between heat production and oxygen consumption. Essentially, this means that REE can be estimated through gas exchange. The volume of oxygen and carbon dioxide are evaluated as follows [16, 17]:

(1) $$\begin{array}{c} {\text{VO}}_{2}=\left(V_{I}\times F_{I}{\text{O}}_{2}\right)-\left(V_{E}\times F_{E}{\text{O}}_{2}\right), \end{array}$$

(2) $$\begin{array}{c} {\text{VCO}}_{2}=\left(V_{E}\times F_{E}{\text{CO}}_{2}\right)-\left(V_{I}\times F_{I}{\text{CO}}_{2}\right). \end{array}$$

The mixing chamber defines one data point every 1∼5 minutes, while 10∼20 minutes are required to assess steady state. In these equations, *V*_*I*_ and *V*_*E*_ are inhalation and exhalation volumes, respectively. *F*_*I*_ and *F*_*E*_ represent the fractional volume of O_2_, CO_2_, and N_2_ in inhalation and exhalation gas mixture, respectively. *V*_*E*_ is known through the gas analyzer, but *V*_*I*_ is unknown. *V*_*I*_ is inferred by using Haldane transformation. It is assumed that *V*_*I*_ × *F*_*I*_N_2_ = *V*_*E*_  × *F*_*E*_N_2_ [18]. Then, *V*_*I*_ is calculated as follows:

(3) $$\begin{array}{c} V_{I}=V_{E}\times F_{E}{\text{N}}_{2}\times F_{I}{\text{N}}_{2}^{-1}. \end{array}$$

This transformation assumes that nitrogen (N) is physiologically inert. Therefore, the volume of inspired nitrogen must equal the volume of expired nitrogen. Thus, VO_2_ and VCO_2_ are calculated as follows:

(4) $$\begin{array}{c} {\text{VO}}_{2}=V_{E}\times \left(F_{I}{\text{O}}_{2}-F_{E}{\text{O}}_{2}\right), \end{array}$$

(5) $$\begin{array}{c} {\text{VCO}}_{2}=V_{E}\times \left(F_{E}{\text{CO}}_{2}-F_{I}{\text{CO}}_{2}\right). \end{array}$$

The Weir equation for VO_2_ and VCO_2_ enables REE to be measured through respiration. The Weir equation is as follows [19]:

(6) $$\begin{array}{c} \left(3.94\;{\text{VO}}_{2}+1.106{\text{VCO}}_{2}\right)1.44-2.17\text{UN}=\text{KCAL}. \end{array}$$

VO_2_, VCO_2_, and UN are volume oxygen, volume carbon dioxide, and urinary nitrogen, respectively. The abbreviated equation does not require 24-hour urinary nitrogen (UN):

(7) $$\begin{array}{c} \left(3.94{\text{VO}}_{2}+1.106{\text{VCO}}_{2}\right)1.44=\text{KCAL}. \end{array}$$

Finally, the RQ value is calculated using the following equations with the VCO_2_ and VO_2_ values [12]:

(8) $$\begin{array}{c} \text{RQ}={\text{VCO}}_{2}\times {\text{VO}}_{2}^{-1}. \end{array}$$

The clinical trial was conducted with the developed device and the above formulas were used.

### 2.3. Clinical Trial

In order to validate the respiratory gas analyzer, we compared the developed device to a commercially available device (Vmax 29, VYAIRE Healthcare, USA). All protocols were approved by the Institutional Review Board at Asan Medical Center, Republic of Korea (S2017-0123-0004).

The clinical trial protocol is as follows [20]. After measuring height and weight, the subject relaxes for at least 10 minutes to maintain steady status. The subject begins measuring exhalation gas using Vmax 29 for 15 minutes. When the measurement is over, the subject rests for 10 minutes. After that, they begin measuring exhalation gas via the developed respiratory gas analyzer for the same amount of time. Finally, the recorded data on VO_2_, VCO_2_, RQ, and REE were used to validate correlations between Vmax 29 and the developed respiratory gas analyzer. Both measurement procedures were conducted with the subject in a supine position. A canopy was used for the Vmax 29, while our developed device was portable with an attached mask.

The subjects included in this study were both men and women from 18 to 40 years old, in a good state of health (i.e., neither physical nor mental defects were detected, as well as respiratory issues). Exclusion criteria were those under the age of 18, or over the age of 40, subjects with respiratory diseases or claustrophobia, and those with physical and/or mental weakness.

## 3. Results

We have developed a portable respiratory gas analyzer. In addition, a clinical trial was conducted in order to validate our device compared to a commercial one, the Vmax 29.

### 3.1. Respiratory Gas Analyzer

The developed respiratory gas analyzer is shown in Figure 2. On the top of the device, there is a handle for carrying the device easily and for supporting the tablet PC when the device is working. Below the handle, the device has a space for storing the tablet PC when the device is not working and a slot with a micro-USB (universal serial bus) pin for putting the tablet PC. As in Figure 2, the device is compact and light-weighted, and thus, it can be used as a portable device. The GUI (graphical user interface) consists of four steps with three pop-up screens and one for displaying measuring data. This pop-up screen is used for putting patient profile, executing calibration process, and alarming to wear the mask. The measurement screen shows oxygen and carbon dioxide level and flow rate in real time and shows calculated VO_2_, VCO_2_, RQ, and REE values every two seconds (see Figure 3).

Calibration is mandatory for the accurate measurement of partial pressures of oxygen and carbon dioxide and volume of breath. As in Figure 4(a), to calibrate oxygen and carbon dioxide levels, a standard gas with the oxygen of 12.33% and carbon dioxide of 2.99% was used. The standard gas container is connected to the oxygen and carbon dioxide sensors. After the gas flows through the sensors for at least 10 minutes, the output values of the oxygen and carbon dioxide sensors were recorded and the sensors were calibrated with these values. When we test the calibrated sensors with the standard gas after a day from the calibration, the output of the oxygen sensor was 12.30% and the output of the carbon dioxide sensor was 3.01%, which is quite accurate. For the calibration of the volume of breath, a certified commercial syringe for volume calibration (3-liter calibration syringe 5530 series, Hans Rudolph, Inc., USA), which freely adjusts the volume flow from 0 to 3000 ml, was used (Figure 4(b)). Since the developed device utilizes a flow sensor, the volume can be calculated by integrating flow rate with time. The volume was measured by varying the total volume of the calibration syringe as 500, 1,000, 1,500, 2,000, 2,500, and 3,000 ml. By using the volume calculated from the flow rate and actual volume flowed, the flow sensor was calibrated. After calibration, the device was tested again six times. Four tests were done at a constant flow rate, and the other two tests were done with changing the flow rate with time.  Figure 5 shows the results. The results show that the error is less than 3% in any tests.

### 3.2. Clinical Result

A photo of the supine position used for clinical trial data collection is shown in Figure 6.

A total of 40 subjects were enrolled in the clinical trial. They consisted of 20 men and 20 women. The age, height, weight, and BMI demographics of each subject are shown in Table 1.

All subjects' mean of age, height, weight, and BMI is 25.40 ± 3.80, 167.20 ± 7.92, 66.69 ± 12.49, and 23.76 ± 3.74, respectively.  Table 2 summarizes all participating subjects.

Figure 7 shows the correlation between Vmax 29 and our developed device; Figures 7(a)∼7(d) show the correlation plots of VCO_2_, VO_2_, RQ, and REE, respectively. The vertical and horizontal axes represent the Vmax 29 and our developed device measured values, respectively. The closer to the baseline is, the greater the equivalence is between the two instruments. The correlation coefficients of VCO_2_, VO_2_, RQ, and REE are 0.86, 0.83, 0.48, and 0.86.

Additionally, Bland-Altman plots were used to compare the performance of the Vmax 29 and our developed device. Bland and Altman introduced the Bland-Altman plot to describe the agreement between two quantitative measurements. They established a method to quantify the agreement between two quantitative measurements by constructing limits of agreement. These statistical limits are calculated by using the mean and the standard deviation of the differences between the two measurements. To check the assumptions of normality of differences and other characteristics, they used a graphical approach.

The resulting graph is a scatter plot *XY*, in which the *Y*-axis shows the difference between the two paired measurements and the *X*-axis represents the average of these measurements. In other words, the difference between the two paired measurements is plotted against the mean of the two measurements. The Bland-Altman plot recommends that 95% of the data points should lie within ±2 SD of the mean difference. This is the most common way to utilize the Bland and Altman plot method, but it is also possible to plot the differences as percentages or ratios instead of the mean. Figures 7(e)∼7(h) show Bland-Altman plots of VCO_2_, VO_2_, RQ, and REE, respectively. Figure 7 shows that most of the VCO_2_, VO_2_, RQ, and REE are within 95% of the significance level.

## 4. Discussion

Throughout this study, the performance of the device we developed highly correlated to that of the Vmax 29, which is a commercial and professional respiratory gas analyzer. However, it is not suitable for personal use due to its large size and price. The respiratory gas analyzer we developed has merits for its lightweight and inexpensiveness.

The results show that the performance of our developed device has a high correlation, greater than 0.8 in VCO_2_, VO_2_, and REE. However, RQ showed a low correlation (0.48). The ratio of VCO_2_ to VO_2_ at rest is 0.7∼0.9. Despite the low correlation of the RQ value, we can see that all the other values are within the correlative range (0.7∼0.9), as shown in Figure 7(c).

A photo of the supine position used for clinical trial data collection is shown in Figure 6. In the same way, measurements were carried out for 15 minutes each, with a 10-minute break time in the middle stage. Since the Vmax 29 uses a canopy that isolates between inner air and external air, the CO_2_, O_2_, and volume flow are measured accurately. However, the system is bulky due to the ventilation system including gas tanks. The developed gas analyzer uses masks instead of canopy for easy portable and easy measurement.

There are several limitations to this study. First, all the subjects were in their 20's and 30's with an active metabolism. This can lead to biased results based upon their young age. Therefore, it would be needed to add older adults and elderly patients, who can truly benefit from such measurements, in future studies. Additionally, all the subjects were of Asian descent and predominantly Korean. A large-scale clinical trial that includes a multitude of ages and races will be necessary to confirm the performance of the developed respiratory gas analyzer.

## 5. Conclusions

We have successfully developed a portable respiratory gas analyzer that displays measurements in real time. The effectiveness of the device was validated through a clinical trial. Although there are limitations to the clinical trial that are dependent on the age and race of the subjects, it is thought that these results can be further proven with a large, more inclusive, clinical trial. The structural problem with the mask can also be improved by developing a new type of mask. These solutions make it possible to develop an improved instrument for more accurate measurement.

The portable respiratory gas analyzer that we developed is more economical and portable than other instruments on the market and is expected to be a suitable model for the home healthcare market.

## Figures and Tables

**Figure 1:** Functional diagram of the respiratory gas analyzer. The flow velocity of the exhaled gas is measured on the mask, and some of it (5%∼10%) is collected using a DC motor. Since the vapor in the collected exhaled gas affects the measurement, the partial pressure of oxygen and carbon dioxide is measured after water is removed using a water trap.

**Figure 2:** The developed portable respiratory gas analyzer, designed for easy measurements. The device is designed to store the tablet PC as well, and the handle serves as a cradle too.

**Figure 3:** The GUI of the developed respiratory gas analyzer. (a) A screen for input patient profile. (b) A screen when the self-calibration is running. (c) A screen for requesting the patient to wear a mask. (d) The measurement screen showing real-time data of oxygen and carbon dioxide level and flow rate and the calculated value of VO_2_, VCO_2_, RQ, and REE every two seconds.

**Figure 4:** Pictures showing the calibration of the developed respiratory gas analyzer. (a) Setup for calibration of the oxygen and carbon dioxide sensors with standard gas containing oxygen levels of 12.33% and carbon dioxide of 2.99%. (b) Setup for calibration of the volume. By using a commercial calibration syringe, calibration was performed with the total volume of 500, 1000, 1500, 2000, 2500, and 3000 ml.

**Figure 5:** The flow rate sensor-based respiratory gas analyzer is accurately calibrated from flow rate to volume flow, which is repeated six times in 500, 1000, 1500, 2000, 2500, and 3000 ml, respectively. (a) When a volume of 500 ml was passed through the gas analyzer, the speed value obtained from the sensor was fitted. To identify dependency, the test is performed four times at similar speeds (A.1∼A.4) and two times at changing the speeds (A.5∼A.6). (b) The average value of under area integration of raw flow rate is fitted at each volume. As a result, the accuracy was obtained with linearity and an error rate of not more than 3%.

**Figure 6:** Clinical trial image. (a) The use of reference equipment (Vmax 29) for validation. (b) Measured using the developed device.

**Figure 7:** Clinical trial results. (a∼d) show the correlation plot of VCO_2_ (*R* = 0.86), VO_2_ (*R* = 0.83), RQ (*R* = 0.48), and REE (*R* = 0.86) between the developed device and Vmax 29, respectively. (e∼h) show Bland and Altman plots of VCO_2_, VO_2_, RQ, and REE, respectively.

**Table 1:** Personal information of the subjects enrolled in this study.

No.	Gender	Age (yr)	Height (cm)	Weight (kg)	BMI (kg/m^2^)
1	Man	24	175	86.0	28.08
2		26	172	74.0	25.01
3		23	172	68.6	23.19
4		24	171	74.9	25.61
5		21	160	53.6	20.94
6		26	179	61.6	19.23
7		29	176	69.2	22.34
8		23	176	82.1	26.50
9		24	177	86.6	27.64
10		23	173	84.3	28.17
11		24	175	74.0	24.16
12		24	173	56.5	18.88
13		23	182	83.0	25.06
14		23	165	77.8	28.58
15		30	174	75.2	24.84
16		24	171	74.3	25.41
17		22	162	62.3	23.74
18		26	162	72.1	27.47
19		27	184	80.2	23.69
20		28	176	76.4	24.66
21	Woman	26	165	59.9	22.00
22		26	163	52.3	19.68
23		27	164	48.9	18.18
24		24	165	51.3	18.84
25		20	161	53.2	20.52
26		24	154	47.3	19.94
27		22	171	74.8	25.58
28		36	160	52.6	20.55
29		23	158	95.3	38.17
30		22	165	56.2	20.64
31		29	165	75.5	27.73
32		21	157	54.7	22.19
33		23	164	56.8	21.12
34		34	169	63.0	22.06
35		37	156	61.7	25.35
36		27	162	67.1	25.57
37		23	154	57.7	24.33
38		24	155	48.9	20.35
39		25	165	58.3	21.41
40		29	160	59.3	23.16

**Table 2:** Summary of participating subjects.

	Age (yr)	Height (cm)	Weight (kg)	BMI (kg/m^2^)
	Mean ± SD	Mean ± SD	Mean ± SD	Mean ± SD
Man	24.70 ± 2.36	172.75 ± 6.38	73.64 ± 9.41	24.66 ± 2.79
Woman	26.10 ± 4.80	161.65 ± 4.84	59.74 ± 11.41	22.87 ± 4.40
Total	25.40 ± 3.80	167.20 ± 7.93	66.69 ± 12.49	23.76 ± 3.74

## Data Availability

The data that support the findings of this study are available from the corresponding author upon request.
